The article "High Mobility Group Box-1 Promotes the Proliferation and Migration of Hepatic Stellate Cells via TLR4-Dependent Signal Pathways of PI3K/Akt and JNK" was retracted in 2019. Reasons: errors in the images; unreliable results or conclusions; concerns about the data; concerns about the images.

# High Mobility Group Box-1 Promotes the Proliferation and Migration of Hepatic Stellate Cells via TLR4-Dependent Signal Pathways of PI3K/Akt and JNK

**DOI:** 10.1371/journal.pone.0064373

**Published:** 2013-05-16

**Authors:** Fu-ping Wang, Lei Li, Jing Li, Ji-yao Wang, Ling-yan Wang, Wei Jiang

**Affiliations:** 1 Department of Gastroenterology, Zhongshan Hospital, Fudan University, Shanghai, China; 2 Department of Gastroenterology, Tongji Hospital, Tongji University, Shanghai, China; 3 Biomedical Research Center, Zhongshan Hospital, Fudan University, Shanghai, China; University of Navarra School of Medicine and Center for Applied Medical Research (CIMA), Spain

## Abstract

**Background:**

The migration of hepatic stellate cells (HSCs) is essential to the hepatic fibrotic response, and recently High-mobility group box 1 (HMGB1) has been shown up-regulated during liver fibrosis. Nevertheless, whether HMGB1 can modulate the proliferation and migration of HSCs is poorly understood, as well as the involved intracellular signaling. In this study, we examined the effect of HMGB1 on proliferation, migration, pro-fibrotic function of HSCs and investigated whether toll-like family of receptor 4 (TLR4) dependent signal pathway is involved in the intracellular signaling regulation.

**Methodology/Principal Findings:**

Modified transwell chamber system to mimic the space of Disse was used to evaluate the migration of human primary HSCs, and the protein expressions of related signal factors were evaluated by western blot. Cell proliferation was analyzed by MTT assay, the pro-fibrotic functions of HSCs by qRT-PCR and ELISA respectively. Recombinant human HMGB1 could significantly promote migration of HSCs under both haptotactic and chemotactic stimulation, especially the latter. Human TLR4 neutralizing antibody could markedly inhibit HMGB1-induced migration of HSCs. HMGB1 could enhance the phosphorylation of JNK and PI3K/Akt, and TLR4 neutralizing antibody inhibited HMGB1-enhanced phosphorylation of JNK and PI3K/Akt and activation of NF-κB. JNK inhibitor (SP600125) and PI3K inhibitor (LY 294002) significantly inhibited HMGB1-induced proliferation and migration of HSCs, and also reduced HMGB1-enhanced related collagen expressions and pro-fibrotic cytokines production.

**Conclusions/Significance:**

HMGB1 could significantly enhance migration of HSCs *in vitro*, and TLR4-dependent JNK and PI3K/Akt signal pathways are involved in the HMGB1-induced proliferation, migration and pro-fibrotic effects of HSCs, which indicates HMGB1 might be an effective target to treat liver fibrosis.

## Introduction

Currently, liver fibrosis caused by chronic liver diseases affects millions of people worldwide. Liver fibrosis, which is characterized by excessive deposition of extracellular matrix (ECM), is the hallmark feature associated with the failure of liver function, irrespective of different aetiological onsets [1], [2]. Therefore, a better understanding of the reversible steps in the fibrotic response may lead to the identification of new therapeutic targets.

The article "High Mobility Group Box-1 Promotes the Proliferation and Migration of Hepatic Stellate Cells via TLR4-Dependent Signal Pathways of PI3K/Akt and JNK" was retracted in 2019. Reasons: errors in the images; unreliable results or conclusions; concerns about the data; concerns about the images.

Hepatic stellate cells (HSCs), which are located in the space of Disse between hepatocytes and sinusoidal endothelium, play a central role in the progression of liver fibrosis. Quiescent HSCs are mainly involved in Vitamin A metabolism, but they may proliferate, produce ECM and even migrate following activation [3]. It is increasingly recognized that HSC migration is essential for fibrosis owing to the observation that during cirrhosis HSCs migrate to and accumulate in fibrotic areas far from their usual location [1], [2], [4]. The motility of HSCs can be influenced by changes in their microenvironment, including extracellular matrix and growth factors [4]. In our previous research, we found transforming growth factor-β1 (TGF-β1) induced the migration and cytoskeletal remodeling of rat HSCs following RhoA activation, and the level of RhoA activation determined the motility of the HSCs [5].

High-mobility group box 1 (HMGB1) protein, originally described as a nuclear nonhistone protein with DNA-binding domains, has been implicated as an important endogenous danger signaling molecule and a potent pro-inflammatory cytokine [6]–[8]. HMGB1 can act as a chemoattractant for fibroblasts, endothelial cells and smooth muscle cells, which suggests that HMGB1 can directly stimulate fibroblast proliferation and participate in fibrogenesis [9], [10]. Recently, HMGB1 has been shown up-regulated during liver fibrosis and can promote the proliferation of HSCs [11]. However, specific extracellular and intracellular signals that regulate the proliferation and migration of HSCs are poorly understood.

Several membrane receptors are implicated in HMGB1 signaling, including the receptor for advanced glycation end-products (RAGE) and members of the toll-like family of receptors (TLRs) [12]. RAGE expression in fibrotic liver is restricted to HSCs and also is up-regulated during cellular activation and transition to myofibroblasts [13]. Silencing RAGE expression by specific siRNA can effectively suppress nuclear factor-kappaB (NF-*κ*B) activity, HSCs activation and ECM deposition in the fibrotic liver [14]. Despite the expression of RAGE is up-regulated in activated HSCs, RAGE stimulation by advanced glycation end products (AGE) does not alter their fibrogenic activation [15]. Therefore, RAGE may not contribute directly to hepatic fibrogenesis. On the other hand, the the activation of HSCs with high expressions of TLR4 is closely associated with the progression of liver fibrosis [16]. Hepatic injury is associated with a barrier deficiency and increased hepatic exposure to bacterial products, and the functional TLR4, not TLR2, is required for hepatic fibrogenesis [17]. TLR4-mutant mice have less liver inflammation and fibrosis than TLR4-wild-type mice following bile duct ligation (BDL) and chronic treatment of carbon tetrachloride (CCl_4_), or thioacetamide [15]. Recently, the release of HMGB1 induced by liver ischemia has been reported to be involved in TLR4-dependent reactive oxygen species production and calcium-mediated signaling [18], and TLR-4 is also involved in HMGB1-induced vascular smooth muscle cells migration [19].So whether the interaction of HMGB1 with TLR4 can play a critical role in hepatic fibrosis and the related mechanism still need further investigation.

The article "High Mobility Group Box-1 Promotes the Proliferation and Migration of Hepatic Stellate Cells via TLR4-Dependent Signal Pathways of PI3K/Akt and JNK" was retracted in 2019. Reasons: errors in the images; unreliable results or conclusions; concerns about the data; concerns about the images.

The ligation of HMGB1 to TLR4 results in the activation of diverse intracellular signaling pathways including Jun N-terminal kinase (JNK), phosphoinositide 3-kinase (PI3K) and its downstream serine/threonine kinase (Akt) [20], [21], whose activation is believed to play a major role in regulating the activation, proliferation and migration of HSCs [5], [22], [23]. And PDGF-mediated proliferation and migration of cultured HSCs are associated with the inhibition of Akt phosphorylation [24]. Activated Akt can phosphorylate a number of proteins including glycogen synthase kinase-3β (GSK-3β), 6-phosphofructo-2-kinase, and inhibitor kappa B (IκB) [25]. The phosphorylation of IκB frees NF-κB and allows it to translocate to the nucleus to bind and subsequently activate target genes [26]. Activation of the transcription factor NF-κB has been demonstrated in activated HSCs [27] and many drugs ameliorate liver fibrosis progression and influence fibrotic functions of HSCs through NF-κB signaling [28]. Based on these findings, the purpose of this study is to investigate whether HMGB1 can induce proliferation and migration of HSCs and whether TLR4-dependent signal pathway is involved in the mechanism.

Here, our results suggest that HMGB1 can significantly stimulate migration of HSCs *in vitro*, and TLR4-dependent JNK and PI3K/Akt signal pathways are involved in the HMGB1-induced proliferation, migration and pro-fibrotic effects of HSCs. To our knowledge, this is the first report on HMGB1- associated HSCs migration. These data further indicates a significant pro-fibrotic function of HMGB1 and its possibility of being an effective target to treat liver fibrosis.

## Materials and Methods

### Ethics Statement

The study protocol was approved by the Research Ethics Committee of Zhongshan Hospital (No. 2010-87) and written informed consent was obtained from each subject.

The article "High Mobility Group Box-1 Promotes the Proliferation and Migration of Hepatic Stellate Cells via TLR4-Dependent Signal Pathways of PI3K/Akt and JNK" was retracted in 2019. Reasons: errors in the images; unreliable results or conclusions; concerns about the data; concerns about the images.

### Regents

Recombinant human HMGB1 was purchased from R&D systems (Minneapolis, MN, USA). Human TLR4 neutralizing antibody was obtained from Invivogen (San Diego, CA, USA). JNK inhibitor (SP600125) was obtained from Sigma-Aldrich (St. Louis, MO, USA), and ConA (10 µg/mL) and PI3K inhibitor (LY 294002) were obtained from Santa Cruz Biotechnology (Santa Cruz, CA, USA). Anti-JNK, anti-phospho-JNK, anti-phospho-PI3K, anti-PI3K, anti-phospho-Akt, anti-Akt, anti-NF-κB, anti- IκB, anti-phospho-IκB and anti-GAPDH antibodies were obtained from Cell Signaling Technology (Beverly, MA, USA).TransAM kit was purchased from Active Motif (Carlsbad, CA, USA) and the NE-PER nuclear and cytoplasmic extraction kit was from Pierce (Rockford, IL). The Annexin V-FITC Apoptosis Detection Kit was obtained from eBioscience (San Diego, CA, USA).

### Preparation of human primary hepatic stellate cells

Human primary HSCs were obtained from liver specimens of patients with hepatic hemangioma who had undergone surgical resections. HSCs were isolated using methods previously described in detail [28]. They were cultured at a concentration of 1×10^5^ cells per well in high glucose Dulbecco's modified Eagle's medium (DMEM, Gibco, Grand Island, NY, USA) containing 20% FCS for 1–2 (quiescent), 3–5 (intermediate), or 7–10 (activated) days as described elsewhere. Cell viability was greater than 90% as assessed by trypan blue exclusion. The purity of the HSCs ranged from 90% to 95% as determined by glial fibrillary acidic protein (GFAP) staining and the typical microscopic appearance of the lipid droplets. On days 1–2, the HSCs were quiescent, round, had abundant lipid droplets, and lacked α-smooth muscle actin (α-SMA) expression. At day 7, the cells had become activated and expressed α-SMA. Cells from days 3–5, which had an intermediate appearance, were chosen for *in vitro* analyses in this study.

### Cell viability assay

The cytotoxicity of HMGB1 toward HSCs was evaluated using a cell viability assay. In brief, after incubation of HSCs with HMGB1 (1–1000 ng/ml), the cells were exposed to 0.4% trypan blue solution for 5 minutes and viewed under a light microscope. Cell viability was defined as the ratio of unstained cells to the total number of cells.

### Cell migration assay

During liver fibrosis, the basement membrane– like matrix is progressively replaced by fibrillar matrix and profibrogenic growth factors, such as PDGF-BB, TGF-β1, EGF, bFGF, and VEGF, which are released by hepatocytes, inflammatory cells, and activated HSCs. In the Boyden chamber system, the upper compartment mimics the normal space of Disse microenvironment, which is mainly comprised of a basement membrane–like matrix (represented by type IV collagen or Matrigel coating of the upper side of the polycarbonate membrane), and the lower compartment mimics inflamed areas of liver microenvironment which is characterized by fibrillar matrix (represented by type I collagen or fibronectin coating of the lower side of the polycarbonate membrane). To delineate different properties of growth factors in facilitating migration of activated HSCs, experiments were performed as follow to test the migratory behavior of cells after direct stimulation in the upper chamber (mimicking HSCs direct stimulation) or in the lower chamber (mimicking chemotactic stimuli from the injured lower compartment).

The article "High Mobility Group Box-1 Promotes the Proliferation and Migration of Hepatic Stellate Cells via TLR4-Dependent Signal Pathways of PI3K/Akt and JNK" was retracted in 2019. Reasons: errors in the images; unreliable results or conclusions; concerns about the data; concerns about the images.

Polyvinyl/pyrrolidone–free polycarbonate membranes with 8 µm pores, which separate the upper and lower wells in a transwell chamber system (Corning, NY, USA), were coated with type IV collagen on the upper side (50 µg/ml) and type I collagen on the lower side (50 µg/ml), as previously described. The bottom wells of the chamber were filled with DMEM, and 2×10^4^ cells/well, which had been serum starved for 24 h, were added into the upper chamber. HMGB1 (1–1000 ng/ml) was added into the upper chamber as a direct haptotactic stimulant, and into the lower chamber as an indirect chemotactic stimulant, to mimic the *in vivo* autocrine and paracrine mechanisms of cytokines respectively. The transwell chamber was incubated at 37°C for 4 h to allow the migration of cells through the membrane into the lower chamber. The migrated cells were stained with Hema3 according to the manufacturer's protocol (Biochemical Sciences Inc., NJ, USA) and counted in six random fields on a phase contrast microscope.

### Western blot

HSCs were washed twice with ice-cold PBS and prepared with RIPA buffer (50 mM Tris-HCl, 150 mM NaCl, 1% Nonidet P-40, 0.5% deoxycholate and 0.1% SDS) containing protease inhibitor mixture (Roche). The samples were separated by SDS-PAGE and then transferred onto a polyvinylidene difluoride membrane (Millipore, Billerica, MA, USA) using SemiDry Transfer Cell (Bio-Rad, Hercules, CA, USA). The polyvinylidene difluoride membrane was blocked with 5% non-fat milk for 3 h followed by incubation with primary antibody in TBST (100 mM Tris–HCl, pH 7.5, 0.9% NaCl, 0.1% Tween 20) overnight at 4°C with gentle shaking: the specific primary antibodies against JNK, p-JNK, PI3K, p-PI3K, Akt, p-Akt, NF-κB, IκB and p-IκB. The blots were incubated with an HRP-conjugated anti-GAPDH antibody (1∶10,000) for 1 h at room temperature. The ratio of each protein to GAPDH was calculated as the relative quantification.

The article "High Mobility Group Box-1 Promotes the Proliferation and Migration of Hepatic Stellate Cells via TLR4-Dependent Signal Pathways of PI3K/Akt and JNK" was retracted in 2019. Reasons: errors in the images; unreliable results or conclusions; concerns about the data; concerns about the images.

### Inhibition experiments

First HSCs, which had been incubated with human TLR4 neutralizing antibody (10 µg/mL) for 1 h, were collected and added into the upper chamber of modified transwell chamber system, and then HMGB1 (100 ng/ml) was added into the upper chamber as a direct haptotactic stimulant or into the lower chamber as an indirect chemotactic stimulant to test whether the TLR4 is involved in HMGB1-induced HSCs migration. Second, TLR4 neutralizing antibody (10 µg/mL) was incubated with human primary HSCs for 1 h, and then HMGB1 (100 ng/ml) was added into the culture medium to determine whether the TLR4 is involved in HMGB1-induced HSCs proliferation and activation of JNK, PI3K/Akt and NF-κB. Third, JNK inhibitor (SP600125, 100 nM) and PI3K inhibitor (LY 294002, 25 mM) were incubated with human primary HSCs for 1 h, and then HMGB1 (100 ng/ml) was added into the culture medium to determine whether the JNK and PI3K/Akt signal pathways are involved in HMGB1-induced HSCs proliferation and pro-fibrotic effects. Finally, HSCs, which had been incubated with SP600125 and LY 294002 at above concentrations for 1 h, were then collected and added into the upper chamber of modified transwell chamber system and HMGB1 (100 ng/ml) was added into the upper chamber or the lower chamber to test whether the JNK and PI3K/Akt signal pathways are involved in HMGB1-induced HSCs migration.

### Determination of NF-*κ*B activity

NF-*κ*B activity was determined using TransAM kit from Active Motif (Carlsbad, CA, USA), according to the manufacturer's instructions. Nuclear and cytosolic fractions were prepared using NE-PER nuclear and cytoplasmic extraction kit from Pierce (Rockford, IL), according to manufacturer's instructions. Briefly, nuclear extract from control and HMGB1-treated HSCs with or without TLR4 neutralizing antibody were added to 96-well plates pre-coated with the oligonucleotide containing NF-*κ*B consensus sequence (5′-GGGACTTTCC-3′). Following incubation at room temperature for 1 h to facilitate the binding, a primary antibody, which recognizes only activated NF-*κ*B/p65, was added to each well. The absorbance was read at 450 nm using a Lab System ELISA plate reader. This assay is specific for NF-*κ*B/p65 activation and more sensitive than electrophoretic mobility shift assay.

### HSCs proliferation assay

The HSCs, trypsinised from the cultures, were resuspended at 1×10^6^ cells/ml and then inoculated into 96-well plates at 1000 cells per well. Cells were incubated with 20 µl methyl thiazolyl tetrazolium for 4 h. After centrifugation, 150 µl dimethyl sulfoxide was added to the precipitate and the absorbance of the enzyme was measured at 490 nm. Cell growth rates (average absorbance of each inhibited group/non-inhibited group) were then calculated. All groups of experiments were performed in triplicate.

The article "High Mobility Group Box-1 Promotes the Proliferation and Migration of Hepatic Stellate Cells via TLR4-Dependent Signal Pathways of PI3K/Akt and JNK" was retracted in 2019. Reasons: errors in the images; unreliable results or conclusions; concerns about the data; concerns about the images.

### HSCs apoptosis assay

To detect early apoptotic changes, staining with Annexin V–fluorescein isothiocyanate (FITC) was used, because of its known high affinity to phosphatidylserine. In the early phases of apoptosis, phosphatidylserine is translocated to the outer layer of the membrane (i.e. the external surface of the cell) and the cell membrane itself remains intact. In contrast to apoptosis, necrosis is accompanied by loss of cell membrane integrity and leakage of cellular constituents into the environment. To distinguish apoptosis and necrosis, propidium iodide, a common dye exclusion test, and annexin V–FITC were used in parallel to show membrane integrity after annexin V–FITC binding to cells. Stained cells were analyzed by FACSCalibur (Becton Dickinson) and FlowJo software 7.6.1 (Tristar, El Segundo, CA, USA).

### Quantitative reverse transcriptase-polymerase chain reaction

Total RNA was extracted using TRIzol (Invitrogen, Carlsbad, CA, USA). Following the manufacturer's instructions, reverse transcription was performed using a PrimeScript RT reagent kit with gDNA Eraser (Takara, Beijing, China) and quantitative real-time PCR conducted with a SYBR reverse transcription-polymerase chain reaction Kit (Takara) using the following conditions: 30 seconds at 95°C, followed by a total of 40 two-temperature cycles (5 seconds at 95°C and 30 seconds at 60°C). Each assay was performed in triplicate. For analysis, the expression of target genes was normalized by the housekeeping gene GAPDH. Based on the ΔΔCt method, relative amounts of mRNA were expressed as 2^−△△Ct^. The primer sequences used were as follows: GAPDH sense 5′-TGTGTCCGTCGTGGATCTGA-3′; GAPDH antisense 5′-TTGCTGT TGAAGTCGCAGGAG-3′; collagen type I alpha 1 (COL1a1) sense 5′-TGCTGGCCCCAAGGGTCCTT-3′; antisense 5′-GGCTGCCAGGACTGCCAGTG-3′; collagen type III alpha 1 (COL3a1) sense 5′-CTTAGAAGCTGATGGGATC-3′; antisense 5′-TTGCCTTGCGTGTTTGT-3′; α-SMA sense 5′-AAGAGCATCCGACACTGCTGAC-3′; antisense 5′-AGCACAGCCT GAATAGCCACATAC-3′.

### Detection of cytokines

The pro-fibrotic of cytokines including TGF-β1, platelet derived growth factor (PDGF)-BB, connective tissue growth factor (CTGF) and epidermal growth factor (EGF) principally produced by HSCs in the supernatant were also evaluated using enzyme-linked immunosorbent assay (ELISA) kits (R&D Systems) according to the manufacturer's instructions.

### Statistical analysis

Results are presented as mean ± standard error of the mean (SEM), in triplicate. Statistical analyses were performed using the GraphPad Software Version 5.01 (CA, USA). Student's *t*-test, one-way ANOVA, χ^2^ test and Pearson's rank correlation were performed as appropriate, and *p* values of less than 0.05 (two-tailed) were considered statistically significant.

The article "High Mobility Group Box-1 Promotes the Proliferation and Migration of Hepatic Stellate Cells via TLR4-Dependent Signal Pathways of PI3K/Akt and JNK" was retracted in 2019. Reasons: errors in the images; unreliable results or conclusions; concerns about the data; concerns about the images.

## Results

### HMGB1 promoted the migration of primary human HSCs by both chemotactic and haptotactic mechanisms

To examine the effects of HMGB1 on the migration of primary human HSCs, we employed the modified Boyden Chamber system mimicing the space of Disse in vivo. To mimic both the autocrine and paracrine activities of cytokines in vivo, HMGB1 was either added to the upper transwell chamber containing the cells (haptotactic stimulation) or to the lower chamber not containing cells (chemotactic stimulation) respectively.

As shown in Figure 1A, chemotactic stimulation with 1 ng/ml HMGB1 significantly enhanced the migration of primary human HSCs, whereas a similar haptotactic effect on their migration occurred at or above 10 ng/ml HMGB1. The motility of primary HSCs was not further enhanced by either chemotactic or haptotactic stimulation with HMGB1 at concentrations higher than 100 ng/ml, suggesting that the pro-migratory effect of HMGB1 on primary HSCs peaked at 100 ng/ml. Therefore, a HMGB1 concentration of 100 ng/ml was chosen as the optimal concentration at which to perform subsequent experiments. Furthermore, at all HMGB1 concentrations, chemotactic stimulation proved to be more effective than haptotactic stimulation in the promotion of HMGB1-induced cell migration (*P*<0.05). Furthermore, HMGB1 did not cause any cytotoxic effects at any concentrations (Figure 1B).

**Figure 1:** HMGB1 promoted the migration of primary human HSCs. (A) HMGB1 was either added to the upper transwell chamber containing the cells (haptotactic stimulation) or to the lower chamber not containing cells (chemotactic stimulation). HMGB1 promoted the migration of primary human HSCs by both chemotactic and haptotactic mechanisms. Data are expressed as the mean ± SEM (n = 6). *P<0.05, compared to 0 ng/ml group; #P<0.05, chemotactic stimulation compared to the haptotactic stimulation in the same concentration. (B) HMGB1 did not cause any cytotoxic effects. Cell viability was detected by trypan blue staining. Data are expressed as mean ± SEM (n = 6).

### HMGB1 induced the activation of JNK and PI3K/Akt through TLR4 signaling in HSCs

Firstly, we found the protein expression of TLR4 elevated after the stimulation of HMGB1 especially at the highest concentration (Figure 2A). To investigate the potential mechanisms for HMGB1 to regulate HSCs migration, we assessed the protein levels of JNK, PI3K/Akt in HSCs after the HMGB1 stimulation. We incubated the primary human HSCs with HMGB1 at different concentrations(0,10,100 ng/mL)for 24 h and detected the protein levels of JNK, PI3K, and Akt and their respective active forms(p-JNK, p-PI3K and p-Akt) by western blot. We found the proteins of p-JNK, p-PI3K and p-Akt on HSCs significantly increased in response to HMGB1 stimulation; however no change of JNK, PI3K, and Akt were detected (Figure 2A).

The article "High Mobility Group Box-1 Promotes the Proliferation and Migration of Hepatic Stellate Cells via TLR4-Dependent Signal Pathways of PI3K/Akt and JNK" was retracted in 2019. Reasons: errors in the images; unreliable results or conclusions; concerns about the data; concerns about the images.

**Figure 2:** HMGB1 induced the activation of JNK and PI3K/Akt through TLR4. (A) Representative of significantly elevated expressions of both TLR4 and active forms of JNK, PI3K/Akt (p-JNK, p-PI3K and p-Akt) in response to HMGB1 stimulation at different concentrations. However no change of JNK, PI3K, and Akt were detected. Relative quantification of the active and total forms of JNK, PI3K, and Akt proteins are presented in the right panel. #p<0.05, compared with 0 ng/ml HMGB1; NS, not significant. (B) After pretreated with TLR4 neutralizing antibody (10 µg/mL) for 1 h, HSCs were cocultured with HMGB1 (100 ng/ml) for 24 h and then HMGB1-enhanced expression of p-JNK, p-PI3K and p-Akt were markedly decreased. Relative quantification of the active and total forms of JNK, PI3K, and Akt proteins are presented in the right panel. *p<0.05, compared with 100 ng/ml HMGB1; NS, not significant.

Secondly, to further investigate the possible involvement of JNK and PI3K/Akt signaling in HMGB1-induced migration of HSCs, we tested the expressions of JNK, p-JNK, PI3K/p-PI3K, and Akt/p-Akt by western blot, when HSCs were pretreated with TLR4 neutralizing antibody (10 µg/mL) for 1 h and then HMGB1 (100 ng/ml) was added into the culture medium for 24 h. As shown in Figure 2B, the pretreatment with TLR4 neutralizing antibody pretreatment markedly decreased HMGB1-enhanced expression of p-JNK, p-PI3K and p-Akt, which indicated HMGB1 could induce the activation of JNK and PI3K/Akt pathways through TLR4 in HSCs.

### TLR4 also took part in HMGB1-induced activation of NF-κB

Increased NF-kB activity has been demonstrated in cell proliferation and NF-kB is retained in the cytoplasm in association with inhibitor protein IkBα [29], [30]. Upon phosphorylation on serine residues, IkBα is degraded allowing NF-kB to translocate to the nucleus and activate transcription of genes responsible for cell growth [26]. Employing western blot analysis, we investigated the effect of TLR-4 neutralizing antibody pretreatment on the levels of constitutively expressed NF-kB protein in HSCs stimulated with HMGB1. As shown in Figure 3A, compared to the HMGB1 stimulation, TLR-4 neutralizing antibody pretreatment resulted in a decrease in NF-kB protein level in the cytosolic as well as nuclear fraction. Notably, a decrease in NF-kB protein level was correlated with a decrease in phospho-IkBα while a concomitant increase in the cytosolic IkBα protein level.

The article "High Mobility Group Box-1 Promotes the Proliferation and Migration of Hepatic Stellate Cells via TLR4-Dependent Signal Pathways of PI3K/Akt and JNK" was retracted in 2019. Reasons: errors in the images; unreliable results or conclusions; concerns about the data; concerns about the images.

**Figure 3:** TLR4 took part in HMGB1-induced activation of NF- κ**B.** A:With or no pretreatment of TLR4 neutralizing antibody, HSCs were stimulated by HMGB1 for 24 h to be analyzed the protein levels of NF-kB, phospho-IkBα and IkBα by western blot. Compared to the HMGB1 stimulation, TLR-4 neutralizing antibody pretreatment resulted in a decrease in NF-kB protein level as well as in phospho-IkBα level, while a concomitant increase in the cytosolic IkBα protein level. *p<0.05, compared with 100 ng/ml HMGB1. B: Effect of HMGB1 with or without TLR4 neutralizing antibody on NF-kB/p65 activity determined by an ELISA-based assay as described in Materials and Methods. *p<0.05, compared with 100 ng/ml HMGB1.

To determine if HMGB1 with or without TLR-4 neutralizing antibody pretreatment induced changes in the levels and /or phosphorylation of NF-kB/p65, the effect of HMGB1 on DNA-binding activity of NF-kB was determined and the results are shown in Figure 3B. The NF-kB activity was enhanced by HMGB1 stimulation, whereas the blockage of TLR-4 significantly inhibited that NF-kB activity enhancement.

### The pathways of TLR4-dependent JNK and PI3K/Akt were involved in HMGB1-induced the proliferation and migration of HSCs

First, to investigate whether PI3K/Akt signaling is involved in HMGB1-induced HSCs proliferation, HSCs pretreated with SP600125 or LY294002 were stimulated with HMGB1 and subsequently subjected to the MTT assay separately to examine their proliferation. The proliferation of HSCs stimulated only with HMGB1 was enhanced to about 200% compared with those without any stimualtion (*P*<0.05). And after pretreated with SP600125 or LY294002, the HSCs proliferation was markedly decreased compared with those stimulated only with HMGB1 (P<0.05) (Figure 4A). Second, pretreated HSCs were added to the upper chamber of modified transwell chamber system and then HMGB1 was either added to upper or the lower transwell chamber respectively exactly like the previous performance. We found the HSCs migration induced by both chemotactic and haptotactic stimulation of 100 ng/ml HMGB1 were markedly inhibited after pre-blockage of JNK or PI3K/Akt signal pathway (Figure 4C). Considering the changes of p-JNK and p-PI3K/p-Akt brought by TLR4 neutralizing antibody, we further incubated HSCs with TLR4 neutralizing antibody ahead of HMGB1 to test HSCs proliferation and migration. The results showed that pre-blockage of TLR4 significantly inhibited HSCs proliferation and migration compared with those stimulated only with HMGB1, which was consistent with the outcomes of JNK and PI3K/Akt inhibitor experiments (Figure 4A & 4C).

The article "High Mobility Group Box-1 Promotes the Proliferation and Migration of Hepatic Stellate Cells via TLR4-Dependent Signal Pathways of PI3K/Akt and JNK" was retracted in 2019. Reasons: errors in the images; unreliable results or conclusions; concerns about the data; concerns about the images.

**Figure 4:** TLR4-dependent JNK and PI3K/Akt were involved in HMGB1-induced HSCs proliferation and migration. A: The proliferation of HSCs pretreated with SP600125 (JNK inhibitor) or LY294002 (PI3K/Akt inhibitor) or TLR4 neutralizing antibody for 1 h was analyzed after their incubations with HMGB1 for 24 h by MTT assay. # *P*<0.05, compared with the HMGB1group. B: The apoptosis of HSCs was analyzed by flow cytometry and Annexin V-FITC^+^PI^-^ represented the HSCs apoptosis as shown in the upper part. The apoptosis percent was calculated and shown by the bar chart. C: After pretreatment with SP600125 (JNK inhibitor) or LY294002 (PI3K/Akt inhibitor) or TLR4 neutralizing antibody, the HSCs migration was significantly inhibited compared with those stimulated only with HMGB1 no matter by haptotactic or chemotactic mechanism. *P<0.05, compared with the HMGB1 group stimulated in the same way (haptotactic or chemotactic stimulation). Data in subfigures A–B are both presented as mean ± SEM (n = 6).

Based on the reports that inhibiting the activation of JNK pathway could accelebrate HSCs apoptosis[31], so we decided to investigate whether the preblockage of TLR4 or JNK or PI3K signalings could affect HSCs apoptosis except for their influence on HSCs proliferation. It turned out that HMGB1 decreased the HSCs apoptosis level slightly whereas the preblockage of TLR4, PI3K/Akt and JNK increased cell apoptosis, all of which had no significant difference (Figure 4B).

Integrated with our previous findings, these results suggest TLR4-dependent JNK and PI3K/Akt signal pathways are involved in HMGB1-induced HSCs proliferation and migration.

### The pathways of TLR4-dependent JNK and PI3K/Akt were also involved the pro-fibrotic effects of HMGB1 on HSCs

To investigate whether JNK and PI3K/Akt signaling are involved in the pro-fibrotic effects of HMGB1 on HSCs, the cells which were pretreated with SP600125 or LY294002 were stimulated with HMGB1 and subsequently subjected to q RT-PCR to test gene expressions including Col I, Col III and α-SMA, and also subjected to ELISA to assess the pro-fibrotic cytokines including TGF-β1, PDGF-BB, CTGF and EGF produced by HSCs in the supernatant. The gene expression of Col I and Col III and pro-fibrotic cytokines production of HMGB1-stimulated HSCs were significantly enhanced compared with those without any stimulation, but when pretreated with SP600125 or LY294002, the pro-fibrotic effects of HSCs aggravated by HMGB1 were markedly decreased (*P*<0.05) (Figure 5). Similarly, whether TLR4 is involved in the pro-fibrotic effects of HMGB1 on HSCs needs further study. And the results of pretreatment with TLR4 neutralizing antibody indicated that preblockage of TLR4 obviously decreased the enhancement of pro-fibrotic effects caused by HMGB1 stimulation, no matter the Col I, Col III and α-SMA expressions or the pro-fibrotic cytokines production.

The article "High Mobility Group Box-1 Promotes the Proliferation and Migration of Hepatic Stellate Cells via TLR4-Dependent Signal Pathways of PI3K/Akt and JNK" was retracted in 2019. Reasons: errors in the images; unreliable results or conclusions; concerns about the data; concerns about the images.

**Figure 5:** TLR4-dependent JNK and PI3K/Akt were involved in HMGB1-induced HSCs pro-fibrotic effects. A: HMGB1 enhanced the level of α-SMA, collagen I, collagen III mRNA in primary human HSCs, whereas SP600125, LY294002 and TLR4 neutralizing antibody decreased the level. α-SMA, collagen I, collagen III/GAPDH were considered as the relative mRNA level. Data are expressed as mean ± SEM (n = 6). #P<0.05, compared with the control group;*P<0.05, compared with the HMGB1-stimulated group. B: HMGB1 enhanced the level of TGF-β1 produced by HSCs, whereas SP600125, LY294002 and TLR4 neutralizing antibody decreased that enhancement markedly. C: HMGB1 enhanced the level of PDGF-BB produced by HSCs, whereas SP600125, LY294002 and TLR4 neutralizing antibody decreased that enhancement markedly D: HMGB1 enhanced the level of CTGF produced by HSCs, whereas SP600125, LY294002 and TLR4 neutralizing antibody decreased that enhancement markedly E: HMGB1 enhanced the level of EGF produced by HSCs, whereas SP600125, LY294002 and TLR4 neutralizing antibody decreased that enhancement markedly Data in subfigures B–E are all presented as mean ± SEM (n = 6). # *P*<0.05, compared with the control group at the same time; * *P*<0.05, compared with the HMGB1 group at the same time.

## Discussion

Liver fibrosis represents a transitional and reversible stage between chronic hepatitis and cirrhosis [1]. During liver fibrogenesis, the normal basement membrane-like matrix, which consists largely of type IV and type VI collagens, can be replaced by fibrillar matrix such as collagens type I and type III. Also, cytokines and reactive oxygen species released from injured cells can directly or indirectly act on HSCs [1]–[3]. The key event during liver fibrosis is that HSCs become activated and transform into myofibroblast–like cells, enabling them to proliferate aggressively, produce large amounts of ECM, migrate in a similar manner to tumor cells, and finally accumulate in injured sites to regulate the fibrotic process [4], [5], [22].

Cell migration usually begins in response to extracellular stimuli such as cytokines, ECM and surrounding cells and may activate transmembrane receptors to promote intracellular signal transduction [4], [8]. During liver fibrosis, the migratory features of activated HSCs are responsible for their accumulation in inflammatory regions to interact with adjacent parenchyma cells and non-parenchyma cells. Our findings confirm that HMGB1 can promote the migration of primary human HSCs through both chemotactic and haptotactic mechanisms, as well as the proliferation of HSCs. Furthermore, chemotactic stimulation is proved to be more effective than haptotactic stimulation in inducing the migration of HSCs, suggesting that HMGB1 exerts its pro-migratory effect through paracrine rather than autocrine mechanisms. HMGB1 can be released from both active secretion of various cells, including activated monocytes/macrophages, neutrophils, and endothelial cells, and passive release of necrotic cells [30], [32]–[34]. Therefore, the migration of HSCs may be regulated primarily by intercellular chemokine activity, and the influence of cell-cell interactions on their migration mechanisms should also be addressed in future researches.

The article "High Mobility Group Box-1 Promotes the Proliferation and Migration of Hepatic Stellate Cells via TLR4-Dependent Signal Pathways of PI3K/Akt and JNK" was retracted in 2019. Reasons: errors in the images; unreliable results or conclusions; concerns about the data; concerns about the images.

TLR4, as a novel receptor for HMGB1, is capable of evoking the immune and inflammatory response through its intra-cellular signal pathways. TLR4 enhances TGF-β signaling and hepatic fibrosis, and LPS-mediated signaling through TLR4 has been identified as key fibrogenic signal in HSCs [35], [36]. PI3K/Akt, which has been shown as activated downstream of TLR4 [37], [38], is critically needed for the regulation of cells growth, migration, and proliferation [22]–[24]. In vivo, inhibition of PI3K signaling inhibits extracellular matrix deposition and reduces expression of profibrogenic factors including TGF-β, tissue inhibitor of metalloproteinase 1 (TIMP-1), and CTGF [23]. In vitro, inhibition of PI3K signaling in HSCs not only decreases the proliferation, collagen expression and several profibrogenic gene expressions of HSCs, but also promotes cell death [39]. However in this experiment, inhibiting PI3K did not increase HSCs apoptosis level, nor did JNK inhibitor. It can be explained by the different HSCs status (intermediate) partly, and why the ability of JNK inhibitor to enhance the HSCs sensitization to induced apoptosis[31] did't display probably is that HMGB1 actually didn't induce apoptosis. Till now,HMGB1 has been found to modulate functions of many cell types, such as human airway epithelial cells, leukemia cells, lung adenocarcinoma cells, through PI3K/Akt signal pathway [40]–[42]. On the other hand, human activated HSCs utilize components of TLR4 signal transduction cascade to stimulate NF-*κ*B and JNK and up-regulate chemokines and adhesion molecules [36]. As to other cell line like Kuffer cells, HMGB1 can induce proinflammatory cytokines production after sever burn injury, largely dependent on TLRs-dependent MAPKs/NF-kB signal pathway[43]. In our previous research, JNK signaling had been shown activated following RhoA activation, which determined the motility of the HSCs [5]. Moreover, activated Akt can phosphorylate IκB, which frees NF-κB to allow it to translocate to the nucleus to bind and subsequently activate target genes [44], and NF-κB activity is essential for PI3K/Akt-induced oncogenic transformation [45]. Thus, it will be interesting to determine whether the signal pathways of JNK and PI3K/Akt are involved in HMGB1-induced HSCs migration via TLR4.

The article "High Mobility Group Box-1 Promotes the Proliferation and Migration of Hepatic Stellate Cells via TLR4-Dependent Signal Pathways of PI3K/Akt and JNK" was retracted in 2019. Reasons: errors in the images; unreliable results or conclusions; concerns about the data; concerns about the images.

First, we found the HSCs migration in response to HMGB1 stimulation was markedly inhibited by pretreatment with TLR4 neutralizing antibody, which indicated TLR4 was involved in HMGB1-induced HSCs migration. Second, we demonstrated that HMGB1-enhanced phosphorylate expressions of JNK, PI3K/Akt and activity of NF-κB in HSCs were significantly suppressed by TLR4 neutralizing antibody, which indicated HMGB1 could induce the activation of JNK and PI3K/Ak through TLR4 in HSCs. Third, by using JNK inhibitor (SP600125) and PI3K inhibitor (LY294002) to block the signal pathway of JNK and PI3K/Akt, we demonstrated that blockage of JNK and PI3K reduced HMGB1-induced activation of NF-κB in HSCs. Fourth, by using modified Boyden Chamber system, HMGB1- induced migration of HSCs were markedly inhibited after pre-blockage of JNK and PI3K/Akt signal pathways. Integrating all these findings, we confirm that TLR4-dependent signal pathways of JNK and PI3K/Akt are involved in HMGB1-induced migration of HSCs. Furthermore, after the pre-treatment with specific inhibitors of JNK and PI3K/Akt, HMGB1-enhanced proliferation and related pro-fibrotic cytokines production of HSCs were markedly inhibited, which indicated the signal pathways of JNK and PI3K/Akt were involved in the pro-fibrotic effects of HMGB1 on HSCs.

Nevertheless, the suppression of HMGB1-induced cells proliferation, migration and pro-fibrotic effects induced by blocking TLR4, JNK and PI3K/Akt signal pathways were often incomplete, indicating other signal pathways might be involved in the regulatory mechanisms. First, TLR4 inhibitor even at much higher concentration could not completely abolish HSCs migration mediated by HMGB1, which could be explained by that other membrane receptors especially RAGE could also participate in this regulatory process [46]. As mentioned previously, RAGE expression in fibrotic livers is restricted to HSCs and its expression is up- regulated during cellular activation and transition to myofibroblasts [13], [14]. Second, ligation of HMGB1 to TLR4 can also activate other intracellular signal pathways besides JNK and PI3K/Akt signal pathway. For instance, MAPK / ERK signaling is involved in the HSCs proliferation and TGF-β1 can mediate the migration of HSCs possibly by Smad2/3 phosphorylation and MAPK pathway [47], [48]. Novo et al. showed that mitochondrial-dependent ROS-mediated activation of ERK and JNK participated in hypoxia-induced migration of HSCs [49]. Our previous study also showed that following RhoA activation TFG-β1 induced the activation of Smad and p38, which determined the motility of the HSCs [5]. Therefore, it is necessary to further explore the intracellular signaling mechanisms underlying the chemotactic action of HMGB1 in HSCs.

The article "High Mobility Group Box-1 Promotes the Proliferation and Migration of Hepatic Stellate Cells via TLR4-Dependent Signal Pathways of PI3K/Akt and JNK" was retracted in 2019. Reasons: errors in the images; unreliable results or conclusions; concerns about the data; concerns about the images.

Taken together, our results have demonstrated that HMGB1 promotes the proliferation and migration of HSCs via TLR4-dependent signal pathways of JNK and PI3K/Akt, which indicates a significant functional role of HMGB1 in the development of liver fibrosis and HMGB1 may be an effective target to treat liver fibrosis. But whether HMGB1 interacts with other TLRs to modulate the functions of HSCs, whether RAGE-mediated signaling also participates in the modulation of HSCs and whether other intracellular signal pathways are involved in HMGB1-induced proliferation and migration of HSCs, require further investigation.
